# Enhanced Adsorption of Zn(II) onto Graphene Oxides Investigated Using Batch and Modeling Techniques

This article has been retracted.

**DOI:** 10.3390/nano8100806

**Published:** 2018-10-09

**Authors:** Min Pan, Guangxue Wu, Chang Liu, Xinxin Lin, Xiaoming Huang

**Affiliations:** 1 Fujian Engineering and Research Center of Rural Sewage Treatment and Water Safety, School of Environmental Science and Engineering, Xiamen University of Technology, Xiamen 361024, China; lin.xinxin@outlook.com; 2 Graduate School at Shenzhen, Tsinghua University, Shenzhen 518055, China; wu.guangxue@sz.tsinghua.edu.cn; 3 College of Environmental Science and Engineering, Anhui Normal University, Wuhu 241002, China; lc2014@ahnu.edu.cn

**Keywords:** graphene oxides, surface complexation modeling, adsorption, Zn(II)

## Abstract

Graphene oxide (GO) was synthesized and employed as an adsorbent for Zn(II) removal from an aqueous solution. The adsorption isotherms showed that Zn(II) adsorption can be better described using the Freundlich model than the Langmuir model. The maximum adsorption capacity of Zn(II) on GO determined using the Langmuir model at pH 7.0 and 293 K was 208.33 mg/g. The calculation of thermodynamic parameters revealed that the process of Zn(II) adsorption on GO was chemisorptions, endothermic, and spontaneous. Kinetic studies indicated that the pseudo-second-order kinetic model showed a better simulation of Zn(II) adsorption than the pseudo-first-order kinetic model. On the basis of surface complexation modeling, the double layer model provided a satisfactory prediction of Zn(II) by inner-sphere surface complexes (for example, SOZn^+^ and SOZnOH species), indicating that the interaction mechanism between Zn(II) and GO was mainly inner-sphere complexation. In terms of reusability, GO could maintain 92.23% of its initial capability after six cycles. These findings indicated that GO was a promising candidate for the immobilization and preconcentration of Zn(II) from aqueous solutions.

## 1. Introduction

With the rapid development of agricultural and industrial activities, massive wastewater caused by heavy metal ions is generated. Increasing attention has been paid to the pollution of heavy metals due to their poisonous effect on organisms even at trace levels, such as cancer, anemia, and intellectual disability [1,2]. Zn can be toxic through the food chain via bio-accumulation [3]. Hence, it is mandatory to decontaminate heavy metal ions to permissible limits (5 mg/L in drinking water according to The World Health Organization). As one of the typical heavy metals, Zn is often found in effluent from mining, smelting, machinery manufacturing, instrumentation, etc. Currently, Zn(II) removal from liquid has been investigated through chemical precipitation, ion exchange, membrane separation, adsorption, and coagulation [3,4,5,6]. Among these methods, the adsorption process is extensively considered as an effective and efficient approach due to its low cost, easy handing, the availability of various adsorbents, and its environment-friendly properties [1]. To date, there has been plenty of literature regarding Zn removal on various adsorbents such as active carbon [7], carbon nano-materials [8], magnetic nanoparticle [9], nano-scale zero-valent iron [10], mineral [4,11], etc. Ggasemi et al. (2015) demonstrated that the maximum adsorption capacity of Zn(II) was only 24.21 mg/g using dioctylphetalate triethylenetetraamine magnetic nanoparticles [9]. Therefore, the development of highly efficient adsorbents for Zn(II) removal was still required, especially for actual application in environmental clean-up operations.

Graphene oxide (GO), as a new two-dimensional carbon-based material, has been widely explored due to its large specific surface area (about 2600 m^2^/g), high mechanical strength (>1060 GPa), and plentiful oxygenous functionalities (e.g., carboxyl, epoxy, and hydroxyl groups) [12,13,14,15]. Thus, GO is deemed to be a promising sorbent for the removal of heavy metal ions [3,16,17,18,19], humic acid [20], radionuclides [14,21,22,23,24], organic dyes [25,26], ammonia [27], etc. Wang (2013) demonstrated that the maximum adsorption capacity of GO was 246 mg/g for Zn(II) [3]. Zhang (2016) also found that the removal efficiency of Zn was 98.07% through GO-based framework composite membranes [16]. However, most research has focused on the adsorption mechanisms by investigating adsorption isotherms and kinetics coupled with the effects of experiment conditions (such as pH, temperature, time, etc.) on adsorption behaviors. Modeling evidence of Zn(II) adsorption onto GO is limited. Surface complexation modeling, as a powerful tool, has been widely applied to fit the adsorption behaviors. In our previous study, the highly efficient adsorption of Pb(II) onto GO was well-simulated by employing surface complexation modeling with SOPb^+^ species and (SO)_2_Pb_2_(OH)_3_^−^ species [28]. Ding et al. (2014), using surface complexation modeling, determined that the sorption performance of GO was attributed to the type and amount of the oxygen-bearing functionalities [29]. However, few studies regarding the prediction of Zn(II) onto GO using surface complexation modeling are currently available.

This study aims to synthesize GO and explore the interaction mechanisms of Zn(II) adsorption on GO subject to analytical techniques (such as X-ray diffraction (XRD), scanning electron microscopy (SEM), transmission electron microscopy (TEM), Fourier transformed infrared (FTIR), X-ray photoelectron spectra (XPS), Raman, and Zeta potential), batch experiments (pH effect, ionic strength effect, kinetic study, and temperature effect), and surface complexation modeling. The key objective of this work is to reveal the fate and transformation of Zn(II) on GO nano-material, which can be considered as a promising absorbent used for the removal of heavy metals in environmental remediation.

## 2. Materials and Methods

### 2.1. Materials

Graphite (<20 μm, 99.99% purity) was purchased from Qingdao Tianhe Graphite Co. Ltd. (Qingdao, China). Concentrated H_2_SO_4_ (98%), KMnO_4_, H_2_O_2_ (37 wt%) and NaNO_3_ were purchased from Sinopharm Chemical Reagent Co. Ltd. (Shanghai, China). The Zn(II) stock solution (50 mg/L) was prepared by dissolving Zn(NO_3_)_2_ in deionized water under ambient conditions and then diluted with deionized water to obtain all the working solutions of Zn(II).

### 2.2. Synthesis and Characterization of GO

The GO was synthesized using the modified Hummers method. Generally, flake graphite was preoxidized by slowly adding 2.0 g flake graphite and 1.5 g NaNO_3_into concentrated H_2_SO_4_ in vigorous stirring and ice-water conditions. Sequentially, the preoxidized graphite was further oxidized by adding 9.0 g of KMnO_4_, and then the suspensions were reacted under room temperature for 5 days. Then, 120 mL 5% of H_2_SO_4_ and H_2_O_2_ solution were added to remove the abundant MnO_4_^−^ ions. Details on the synthesis of GO are described in our previous research [28].

The morphology of GO was evaluated using a scanning electron microscope (SEM JEOL-6060SEM, JEOL Ltd., Tokyo, Japan) and a transmission electron microscope (TEM JEM-2010 JEOL Ltd., Tokyo, Japan). The FTIR spectra of GO were identified using Bruker Vector 22 (Bruker, Madison, WI, USA). The XPS spectrum was conducted using a thermo ESCALAB 250 electron spectrometer (Thermo Fisher Scientific, Waltham, MA, USA). GO was examined using the XRD analysis with a Rapid-II powder diffractometer (D/RAPID II, Rigaku, Tokyo, Japan) with CuKa radiation. The XRD pattern was taken in the range of 5–70° at a scan speed of 4°/min. Raman spectroscopy was carried out on the LabRam HR Raman spectrometer (Horiba, Paris, France) with an Ar^+^ laser. The zeta potential of GO was confirmed using a zeta meter (Nano ZS Zetasizer, Malvern, UK).

### 2.3. Batch Adsorption Experiments

To investigate the adsorption characteristic of Zn(II) on GO, a batch technique in polyethylene centrifugal tubes under room temperature conditions was conducted. Specifically, the GO solution was mixed with a freshly prepared Zn(II) solution in the presence of 0.01 M NaClO_4_ solution. The pH values in the aqueous solution were regulated by adding 0.01–1.0 mol/L HClO_4_ or NaOH solution drop by drop. After being centrifuged at 6000 rpm for 30 min, the supernatant was used to determine the Zn(II) concentration using atomic absorption spectroscopy (AA-6300C, Shimadzu, Japan). All the experimental data obtained in this study were the mean values of duplicate or triplicate measurements and the relative error was <5%. The equilibrium adsorptive capacity was calculated using the following equation:

(1) $$q_{t}=\frac{(C_{0}-C_{t})v}{m}\;$$

where *q_t_* is the adsorptive capacity at time *t*, mg/g; *C*_0_ and *C_t_* (mg/L) are the Zn(II) concentration in the aqueous solution at the beginning and time *t*, respectively; *v* is the volume of the solution, L; and *m* is the mass of the adsorbent, g.

### 2.4. Surface Complexation Modeling

The adsorption of Zn(II) on GO is simulated using the diffuse layer model (DLM) of surface complexation modeling with the help of the FITEQL v 4.0 code [28,30]. The values of the protonation and deprotonation constants (logK^+^ and logK^−^) are described using Equations (2) and (3), respectively:

(2) $$\mathrm{SOH}+H^{+}={\mathrm{SOH}}_{2}{}^{+}{\mathrm{logK}}_{1}{}^{+}{=\log([\mathrm{SOH}}_{2}{}^{+}{]/[\mathrm{SOH}][H}^{+}])\;$$

(3) $${\mathrm{SOH}=\mathrm{SO}}^{-}+H^{+}\log K_{2}{}^{-}=\log([SO^{-}][H^{+}]/[\mathrm{SOH}])\;$$

where SOH is represented as the amphoteric surface groups on GO. The values of logK^+^ and logK^−^ were cited from the previous studies. In the existence of 0.01 mol/L NaClO_4_ solution, the surface complexation reactions are expressed as Equations (4) and (5):

(4) $$\mathrm{SOH}+Zn^{2+}=SOZn^{+}+H^{+}\log K_{3}=\log([SOZn^{+}][H^{+}]/[SOH][Zn^{2+}])\;$$

(5) $$SOH+Zn^{2}{}^{+}+H_{2}O=SOZnOH+2H^{+}\log K_{4}=\log([SOZnOH]{\left[H^{+}\right]}^{2}/[SOH][Zn^{2+}])\;$$

The equilibrium constants (logK values) can be received by optimizing the simulated results with the adsorption data.

## 3. Results and Discussion

### 3.1. Characterization

Figure 1A,B show the observation from the SEM and TEM techniques of GO, respectively. The wrinkled, aggregated, and thin nanosheets were clearly observed, which corresponded with the previous study [29]. According to the TEM images of GO, the mean thickness of GO was near 2.5 nm (Figure 1B). As shown in the FTIR spectrum (Figure 1C), the peaks at ~1045, 1450, 1630, 1720, and 3440 cm^−1^ contributed to the stretching vibration of the C–O–C, C=O, C=C, COOH and COH groups, respectively [31]. XPS, as a powerful tool, can characterize the chemical constituents and electronic structures of GO. Figure 1D shows the deconvolution of high-resolution O 1s XPS spectra of GO. The binding energy of O 1s XPS at 531.25, 532.48, 533.02, and 533.45 eV can be indexed to C=O, C–O–C, C–OH and adsorbed H_2_O (chemisorbed/intercalated adsorbed water molecules), respectively. The findings from the XPS analysis illustrated that the GO sheets were decorated with plentiful oxygenic functionalities (such as hydroxyl, epoxy, carboxyl, and carbonyl groups) [32]. Figure 1E illustrates the XRD pattern of GO. Ragubanshi et al. (2017) found that the diffraction peak of pure graphite was appropriately 2θ = 26.58° [33]. One can see that only one weak diffraction peak at 2θ = 10.66° was shown, which corresponded to the GO nanosheets and was attributed to the (002) plane. The absence of a peak of pure graphite suggested that an excellent separation and high quality of GO was produced. The interplanar spacing of GO was estimated to be 0.945 nm, which was consistent with previous work [34]. Raman spectroscopy of GO indicated the D-band at 1350 cm^−1^ and the G-band at 1590 cm^−1^ (Figure 1F). It is well-known that the D-band reflects disorders and local defects while the G-band is related to the vibrations of SP^2^ of carbon atoms in a graphitic 2D hexagonal lattice [33,35]. The *I*_D_/*I*_G_ ratio was calculated as 0.91, implying less disorder and defect concentration and more perfect aromatic structure in GO. 

### 3.2. Effect of pH and Ionic Strength

Figure 2A shows the effect of pH on Zn(II) adsorption onto GO by altering the pH value from 2.0 to 10.0. It clearly demonstrates that Zn(II) adsorption rapidly increased with an increase in the pH from 2.0 to 7.0, preserved at a high-degree sorption at pH 7.0–8.0, and slightly decreased from pH 8.0 to 10.0. The adsorption was determined to be a pH-dependent process. In Figure 2B, the main species of Zn in liquid were Zn^2+^ species at pH < 8.5, Zn(OH)_2_ (s) species at pH of 8.5–9.5, Zn(OH)_3_^−^ species at pH 11.0–11.5, and Zn(OH)_4_^2−^ at pH > 12.5. Based on the zeta potential in Figure 2C, GO was negatively charged at pH > 2.0. Thus, the increasing adsorption of Zn on GO at pH 2.0–7.0 could be attributed to the electrostatic attraction between positive Zn^2+^ and negatively charged GO. The significant Zn(II) removal percentage at pH 7.0–8.0 could be attributed to simultaneous precipitation Zn(OH)_2_(s), which was in accordance with the previous study [3]. At pH > 8.0, the electrostatic repulsion between negatively charged GO and Zn(OH)_3_^−^ species and Zn(OH)_4_^2−^ species resulted in a slight reduction in Zn(II) adsorption onto GO.

Figure 2A indicates the influence ionic strength on the adsorption of Zn(II) onto GO with 0.001, 0.01 and 0.1 mol/L NaClO_4_ presented. When the pH value was lower than 4, the removal efficiencies of Zn(II) were slightly increased with the NaClO_4_ concentrations increased. When the pH value was higher than 4, the changes in the removal efficiencies of Zn(II) could be negligible with the NaClO_4_ concentrations increasing. Wang et al. (2013) stated that a foreign ion may affect the affinity to the surface of GO [3]. Weng et al. (2004) found that a foreign ion may influence the electrical double layer structure and then impact the binding of the adsorption species [36]. However, Tan et al. (2017) declared that the sorption of Cu^2+^ on GO changed slightly by increasing Cl^−^ (from 0.01 M to 0.1 M) [17]. Liu et al. (2013) demonstrated that monovalent anions showed a negligible impact on Co(II) adsorption onto carbon nanotube-hydroxyapatite composites [37], which is consistent with the result obtained in this study. Previous studies proved that ionic strength mainly took charge of the outer-sphere surface complexation and ion exchange, whereas ionic strength showed no impact on inner-sphere surface complexation [31]. Therefore, inner-sphere surface complexation decided the adsorption process of Zn(II) on GO over a wide pH range.

### 3.3. Adsorption Isotherms

The adsorption isotherms of Zn(II) adsorption on GO were simulated using the Langmuir and Freundlich models, which are described as Equations (6) and (7):

(6) $$\frac{C_{e}}{q_{e}}=\frac{1}{q_{m}}C_{e}+\frac{1}{q_{m}k}\;$$

(7) $$\ln q_{e}=\ln K_{f}+\frac{1}{n}\ln C_{e}\;$$

where *C_e_* is the equilibrium Zn(II) concentration in the aqueous solution (mg/L); *q_e_* and *q_m_* refer to the equilibrium adsorption capacity on the adsorbent and the maximum adsorption capacity, respectively (mg/g). The values of k (L/mg) and K_f_ (mg/g) are the adsorption constants of the Langmuir and Freundlich models, respectively. 

By calculating the slope and intercept of the linear plots, the relative parameters of the Langmuir and Freundlich models obtained are exhibited in Table 1. Due to the high correlation coefficients (R^2^ > 0.9272), these two models were sustainably employed to fit the experimental results in this study. In Figure 3, it is clearly observed that the behaviors of Zn(II) sorption onto GO can be better simulated using the Freundlich model with correlation coefficients higher than 0.998 than Langmuir model with correlation coefficients lower than 0.943 in three different temperatures, indicating the adsorption conducted on a structurally heterogeneous sorbent [38]. The *q_m_* of Zn(II) on GO counted using the Langmuir model was 208.33 mg/g at 293 K (Table 1), which was higher than other nano-scale sorbents such as: dioctylphetalate trithylenetetraamine magnetic nanoparticle (24.21 mg/g) [9], nZVI (20.00 mg/g) [7], nanostructured birnessite-type manganese oxide and birnessite/carbon nanotubes (HB/CNTs) (89.50 mg/g) [8]. It was also higher than in other research on GO for Zn(II) removal, for example 73 mg/g of GO prepared using amorphous graphite [39] and 88.12 mg/g of GO prepared using glycine, EDC and NHS [40]. Moreover, the *q_m_* values increased from 208.33 mg/g to 211.42 mg/g with the temperature increasing from 293 K to 313 K (Table 1), indicating that higher temperature promoted a higher adsorption capacity of Zn(II) on GO.

### 3.4. Thermodynamic Parameters

Thermodynamic parameters involving Gibbs free energy change (ΔG^0^), enthalpy change (ΔH^0^), and entropy change (ΔS^0^) are determined by the temperature dependent adsorption isotherms according to the following Equations (8)–(10):

(8) $$K_{d}=\frac{q_{e}}{C_{e}}\;$$

(9) $$\Delta G^{0}=-RT\ln K_{d}\;$$

(10) $$\ln K_{d}=-\frac{\Delta H^{0}}{RT}+\frac{\Delta S^{0}}{R}\;$$

where *K_d_* is the distribution coefficient, mL/g. ΔH^0^ and ΔS^0^ can be obtained by calculating the liner constants for the plot of ln*K_d_* versus 1/*T* (Figure 4). The minus values of ΔG^0^ implied that the behavior of Zn(II) adsorption on GO was a thermodynamically favorable and spontaneous process. The magnitudes of ΔG^0^ reduced from −26.23 kJ/mol to −28.84 kJ/mol coupled with an increase in temperature from 293 to 313 K (Table 2), implying that higher temperatures favored more energetic adsorption. As the value of ΔH^0^ was positive (12.00 kJ/mol), the adsorption of Zn(II) on GO was an endothermic process. With the value of ΔS^0^ (130 J/mol/K) being higher than zero, the extent of randomness was revealed to rise at the solid-solution interface during the sorption process of Zn(II) on GO. It also demonstrated that increasing temperature benefited the spontaneous proceeding of adsorption behaviors.

### 3.5. Adsorption Kinetics

The transient behavior of Zn(II) adsorption is fitted using two typical kinetic models, which are expressed as:

(11) $$\mathrm{Pseudo}\;\mathrm{first}\text{-}\mathrm{order}\;\mathrm{equation}:\;\ln(q_{e}-q_{t})=\ln q_{e}-k_{1}t\;$$

(12) $$\mathrm{Pseudo}\;\mathrm{second}\text{-}\mathrm{order}\;\mathrm{equation}:\;\frac{t}{q_{t}}=\frac{1}{k_{2}q_{e}{}^{2}}+\frac{t}{q_{e}}\;$$

where k_1_ and k_2_ are the respective rate constants (g/(mg h)).

Figure 5 shows the adsorption kinetics of Zn(II) adsorption on GO at 293 K. One can see that the adsorption of Zn(II) on GO rapidly rose up to 75.9% with the reaction time increasing within 3 h. It should be mentioned here that the low removal percentage obtained was mainly due to the low m/v ratio of 0.12 g/L applied in this study. After 6 h, the adsorption removal efficiency of Zn(II) was slightly increased to 78.86%. Comparing the kinetic results of these two kinetic models, the pseudo-second-order model can describe the adsorption kinetic of Zn on GO with higher correlation coefficients (R^2^ > 0.999) very well (Table 3). The adsorption behavior was determined to be chemisorption [28]. Moreover, the adsorption capacity in the theoretical evaluation at equilibrium (167.50 mg/g at 293 K) counted using the pseudo-second-order model was quite close to the adsorption capacity at equilibrium gained from the actual experiment (166.84 mg/g at 293 K). Moreover, the values of *q_e_* rose from 167.5 mg/g to 174.83 mg/g with the temperature increasing from 293 K to 313 K, which corresponded with the findings obtained above. The kinetic data obtained in this study are also consistent with other research demonstrating that the pseudo-second-order model can simulate the kinetics of heavy metals sorption on GO well [28,32,41].

### 3.6. Surface Complexation Modeling

By optimizing the simulated data under various pH cultures, the equilibrium constants obtained from the surface complexation modeling are exhibited in Table 4. As shown in Figure 6, Zn(II) sorption on GO in pH-dependent conditions are satisfactorily fitted by applying DLM with mononuclear and monodentate complexes, SOZn^+^ species and SOZnOH species. It is clearly observed that the main adsorption species was SOZn^+^ species at pH < 4, and the main SOZnOH species charged the adsorption of Zn(II) on GO at pH > 4. The findings from the surface complexation modeling suggested that the sorption of Zn(II) on GO was mainly inner-sphere surface complexation, which corresponded with the findings of the ionic strength adsorption experiments.

### 3.7. Regeneration and Reusability

The repeated availability of GO after desorption by using 0.1 M HCl as an elution agent was investigated. As shown in Figure 7, the adsorption capacity of Zn(II) on GO was slightly reduced. It clearly demonstrates that after three cycles of adsorption-desorption the value of the adsorption capacity of Zn(II) changed from 166.83 mg/g to 164.76 mg/g (appropriate 98.76% of GO regenerated). After six cycles, the adsorption capacity of Zn(II) was 153.84 mg/g, which counted for 92.23% of the initial capacity of the GO. Guo et al. (2017) obtained 86% of the initial adsorption capacity of l-arginine modified magnetic adsorbent after five cycles of adsorption-regeneration on Zn(II) using a 6 mol/L HCl solution (the maximum adsorption capacity was 150.4 mg/g) [42]. Liu et al. (2017) found 90% of the initial Zn(II) removal capacity using nanostructured birnessite-type manganese oxide and birnessite/carbon nanotubes (HB/CNTs) (the maximum adsorption capacity was 89.5 mg/g) [43]. As a whole, the results here demonstrated that GO has satisfactory reuse potential and excellent regeneration performance with a highly efficient adsorption capacity for Zn(II) removal from aqueous solutions, which corresponded with the previous study [3].

## 4. Conclusions

Based on various characterization techniques, plentiful oxygenic functionalities were presented on the surface of GO, which contributed to the highly efficient sorption of Zn(II). The sorption of Zn(II) on GO was irrelevant with ionic strength, revealing that the inner-sphere surface complexation dominated Zn(II) adsorption. According to the Langmuir model, the maximum adsorption capacity of GO for Zn(II) was 208.33 mg/g at pH 7.0 and 293 K. Thermodynamic parameters determined that the adsorption process of Zn(II) on GO was endothermic and spontaneous. The fitting findings of the surface complexation modeling suggested that pH-dependent sorption of Zn(II) on GO can be satisfactorily fitted using DLM with mononuclear and monodentate complexes, SOZn^+^ species and SOZnOH species, at a lower and higher pH, respectively. The findings of this study showed that GO has a potential use in heavy metal removal from aqueous solutions.

## Figures and Tables

**Figure 1:** Characterization of GO ((**A**) SEM image; (**B**) TEM image; (**C**) FTIR spectrum; (**D**) XPS; (**E**) XRD; (**F**) Raman).

**Figure 2:** (**A**) Effect of pH on Zn(II) adsorption onto GO in the presence of 0.001, 0.01, and 0.1 mol/L NaClO_4_; (**B**) Distribution of Zn(II) species in aqueous solution (*C*_0_ = 10 mg/L, m/v = 0.12 g/L, *t* = 24 h, *T* = 293 K); (**C**) Zeta potential of GO dispersion as a function of pH value.

**Figure 3:** (**A**) Langmuir isotherm plots of Zn(II) adsorption on GO; (**B**) The Freundlich isotherm plots of Zn(II) adsorption on GO.

**Figure 4:** Plots of ln*K_d_* vs. 1/*T*.

**Figure 5:** Adsorption kinetics of Zn(II) on GO (*C*_0_ = 25 mg/L, m/v = 0.12 g/L, I = 0.01 mol/L NaClO_4_, *T* = 293 K).

**Figure 6:** The fitted results of surface complexation modeling of Zn(II) on GO at different pH levels.

**Figure 7:** Adsorption-desorption cycles of Zn(II) on GO nanosheets (*C*_0_ = 10 mg/L, m/v = 0.12 g/L, I = 0.01 mol/L NaClO_4_, *T* = 293 K).

**Table 1:** Relative parameters of the Langmuir and Frenudlich isotherm models.

Isotherm Models	Parameters	*T* = 293 K	*T* = 303 K	*T* = 313 K
Langmuir	*q_m_* (mg/g)	208.33	210.97	211.42
	K (L/mg)	0.8727	1.0085	1.1537
	R^2^	0.9096	0.9219	0.9196
Frenudlich	*ln*K_f_ (mg^1−*n*^·L*^n^*/g)	4.3837	4.4883	4.5721
	1/*n*	0.6226	0.6313	0.6321
	R^2^	0.9991	0.9990	0.9991

**Table 2:** Thermodynamic parameters for the adsorption of Zn(II) on GO.

*T* (K)	ΔG^0^ (kJ/mol)	ΔS^0^ (J/mol/K)	ΔH^0^ (kJ/mol)
293	−26.23	130	12.00
303	−27.52		
313	−28.84		

**Table 3:** Kinetic parameters of Zn(II) adsorption on GO.

Kinetic Models	Parameters	*T* = 293 K	*T* = 303 K	*T* = 313 K
Pseudo first-order	*q_e_* (mg/g)	78.16	96.75	92.12
	k_1_ (h^−1^)	0.2947	0.3328	0.292
	R^2^	0.7486	0.6888	0.7688
Pseudo second-order	*q_e_* (mg/g)	167.50	169.78	174.83
	k_2_ (g/mg h)	0.015	0.014	0.018
	R^2^	0.9994	0.9991	0.9992

**Table 4:** Theoptimized parameters of surface complexation modeling for Zn(II) adsorption on GO.

Equations	LogK
Protonation and deprotonation	
SOH + H^+^ = SOH_2_^+^	4.52
SOH = SO^−^ + H^+^	−7.88
Surface complexation modeling	
SOH + Zn^2+^ = SOZn^+^ + H^+^	3.48
SOH + Zn^2+^ + H_2_O = SOZnOH + 2H^+^	−8.64
